# Tripartite Evolutionary Game Analysis of Financial Support for Science-Tech Enterprises' Innovation with Government Participation

**DOI:** 10.1155/2022/5207003

**Published:** 2022-04-30

**Authors:** Wei Liu, Yang Liu, Jun Gu, Jing Zhao, Rong Zhang

**Affiliations:** ^1^Business College of Beijing Union University, Beijing 100025, China; ^2^Kunming University, Kunming, Yunnan 650214, China

## Abstract

In this study, we use a tripartite evolutionary game model to analyze the financial support for science-tech enterprises' innovation with government participation. Based on the game model, the study uses replication dynamics to analyze the stability of evolutionary trajectory in the eight scenarios of enterprises, the government, and the financial institutes. Then, we discuss the effect of the reputation multiplier, the efficiency of firms' innovation output, and the positive socio-economic externalities multiplier by simulation as the important innovative points in this study. The study draws the following conclusions: (1) enterprises will choose high R&D intensity instead of low R&D intensity if the output of former exceeds that of the latter, (2) enterprises' R&D output is closely related to the strategy choices of the government and financial institutes, and (3) enterprises can attract government subsidy by boosting economic and social externalities. The government subsidies to enterprises with high R&D intensity will improve the innovation output by the innovation investment and reputation multiplier. So, the government can implement subsidy policy to boost high-intensive R&D activity. Financial institutes' strategy choice between equity investment and debt investment is influenced by investment yield difference and can influence enterprises' R&D intensity choices.

## 1. Introduction

Intensive innovation is an effective way for companies to improve their core competitiveness [1] (Frambach and Schillewaert) and is a core driver of high quality development. R&D intensity is the key to corporate innovation, and the strategic choice of R&D intensity by companies is mainly based on a cost-benefit analysis. The main source of funding for corporate innovation is internal and external financing, where external financing is constrained by the high risk of innovation projects, credit asymmetry, opportunism, and adverse selection [2, 3] (Brown et al.). Financial institutes disagree on firms' return on investment requirements [4] (Hall, 2002) and intensify financing constraints. Financial institutes' capital investment is considered beneficial to firms' R&D activities [5–7] (Fryges et al.), while higher financing costs arising from financing constraints reduce firms' willingness to invest in R&D, thus reducing firms' willingness to innovate. Due to the positive externalities of technological innovation, governments are active promoters of firm innovation [8] (Yu et al.). A series of initiatives, including financial subsidies, can alleviate the financing constraints and stimulate firms to invest in innovation [9] (Zhou). On the one hand, government subsidies provide good investment signals for equity investment institutions [10–12] (Howell et al.), which is a disguised endorsement of firms' credit and R&D capabilities. On the contrary, government subsidies can reduce the cost of enterprise loan financing by the signal effect. Therefore, it is necessary for governments to understand how firms make choices about R&D intensity and how financial institutes make choices about loans or investment in R&D projects. Thus, government can influence the strategic choices of firms and financial institutes through subsidy policies.

Government subsidies provide the impetus for the development of enterprise innovation, enterprises are the subjects of innovation, and financial institutes provide financial services and financial support for enterprise innovation. Changes in the strategic choices of any of the participants in corporate innovation will lead to corresponding changes in stakeholder response strategies, both in terms of the continuous improvement of information structures and the adjustment of the rational level of multiple participants. There are a lot of research studies on enterprises' R&D strategy, financial institutes' investment strategy, and government subsidy policy. However, there is a lack of analysis that puts the three players in a comprehensive game framework. This study is based on this theoretical framework to introduce enterprises, financial institutes, and government into a comprehensive game in which enterprises choose high or low R&D intensity; financial institutes choose equity or debt investment, while the government chooses whether to provide subsidy. The government's subsidy policy, enterprises' R&D intensity choice, and financial institutions' investment structure influence each other. Therefore, the government can attract enterprises to choose high R&D intensity strategy and financial institutes to make equity investment by adjusting its subsidy policy.

The main innovations of this study are as follows:

1. Current research has focused on measuring risk-sharing ratios among financial institutes [13, 14] and lacks a holistic analysis of the behavior of governments, financial institutes and firms, and their interactions. However, examine the different strategic options and possible interactions between key players. Most previous research has only two players in the game framework without considering the function of government participating. The framework of this study is more complex with reality. The analysis focuses on the different strategic choices and possible interactions of firms, financial institutes, and governments in the process of obtaining external finance for firms with different R&D intensities. It draws some interesting conclusions.
2. Existing studies point out that government financial subsidies for business innovation vary across different types of enterprises [15]. The firms' R&D intensity has an impact on the effectiveness of government intervention. However, we find that the reputation multiplier of government subsidies also has the effect on firm innovation and the choice of investment approach by financial institutes. We also find that firms' innovation efficiency and strategy game affect the investment approach of financial institutes and the choice of government financial support, which in turn affects firms' financing costs.
3. Another possible contribution of this study is to explore how the efficiency of firms' innovation output and the positive socio-economic externalities generated by innovation impact on government and financial support decisions.

The remainder of this study is structured as follows.  Section 2 briefly reviews the existing research on financial support for science-tech enterprises and evolutionary games and presents the literature gaps.  Section 3 constructs a three-party evolutionary game model among SMEs, financial institutes, and government.  Section 4 discusses the ESS of the tripartite game between the government, the financial institutes, and SMEs.  Section 5 presents the numerical simulation result of the evolutionary game model, which discusses the effect of incentive-related parameters on the results.  Section 6 provides discussion of evolutionary results and policy implications.

## 2. Literature Review

This study briefly reviews the literature on financial support for science-tech enterprises and evolutionary game models with the above objectives.

### 2.1. Financial Support for Science-Tech Enterprises

Through numerous studies, scholars have generally concluded that financing constraints have a negative impact on enterprises' R&D and innovation activities [16, 17] (Hottenrott et al.). Different scholars have conducted empirical studies using data from countries such as Germany, France, Spain, and Uruguay and have come to the consistent conclusion that financial support can be effective in stimulating enterprises' R&D investment [18–21] (Almus et al.). Some scholars studied the function of finance support to enterprise science-tech innovation through different channels. Abobal and Garda believed that technological innovation needs capital input such as bank loans [21]. Saint-Paul proposed financial development promotes technological progress by allowing economic entities to use technologies with greater risks but higher levels of productivity [22]. Luong et al. used firm-level data across 26 non-U.S. economies between 2000 and 2010 to show that foreign institutional ownership has a positive and causal effect on firm innovation [23]. Menezes and Pereira found financial product innovation speeds up technological innovation [15]. Kim et al. found that capital market financing could promote technological innovation of enterprises more than bank loans [24]. Research in China suggests that government and market forces need to work together to promote financial support for enterprises' innovation processes [25] (Gong et al.).

In the past few years, the effect of government subsidies on the external investors funding the enterprises' innovation has attracted significant scholarly attention. The government expects to stimulate R&D activities through direct subsidies. Sabrinaconduct that government subsidies have a positive effect on corporate patents [10]. Feldman & Kelley argue that companies that receive R&D subsidies are recognized by the government and send a signal that they are innovative and can attract more investment [26]. The idea is that companies that receive R&D grants are recognized by the government and send a signal that they are innovative, which can attract more investment [12, 27, 28] (Meuleman et al.). However, the inevitable “rent-seeking behavior” can lead to resource misallocation due to government subsidies [29] (Lemer) and distortions in enterprises' competitive behavior [30] (Guellec et al.) and distortions in the competitive behavior of enterprises. Chinese scholars have also demonstrated the positive effects of government subsidies on corporate R&D based on empirical evidence from China. For example, Liu et al. found that government subsidies stimulate enterprises' R&D investment by using data on high-tech enterprises in Jiangsu [31].

### 2.2. Evolutionary Game

The central concepts of evolutionary game theory are evolutionary stable strategies and replicator dynamics, arguing that a group's decisions can be achieved through dynamic behaviors such as imitation, communication, and learning between individuals, while having highly adaptive strategies. Strategies that are highly adaptive are more likely to be imitated by other participants; otherwise, these strategies are eliminated. The theory is an important mathematical tool because it is based on finite theory and finite information and is closer to reality.

In recent years, evolutionary games have rapidly developed into an active area of research in the socio-economic field and are an increasingly popular approach in the study of corporate innovation. Yang et al. developed an evolutionary game model between government, enterprises, universities, and research institutions to explore the mechanisms of intellectual property cooperation [32]. Han et al. used a game model to analyze the effect of cluster informal contracts on innovation cooperation among cluster enterprises and the impact of informal contracts on innovation cooperation among cluster enterprises [33]. Shen used evolutionary game theory to study firm decision-making behavior during open innovation [34]. The impact of heterogeneous structures on the evolution of innovation behavior has been discussed based on scale-free networks [35, 36] (Ma et al.; Su et al.). Some literature use the evolutionary game method to study the optimal government subsidy. For example, Meng and Zhao discussed the optimal subsidy that can promote the system to reach the ideal state by constructing the evolutionary game model between manufacturers and remanufacturers [37] (Meng and Zhao). Bi Peng and Chen used evolutionary game theory to study the cooperative innovation of key common technologies of the two equipment manufacturing enterprises, respectively, constructed an evolutionary game model with or without government macrocontrol, analyzed the key factors affecting the stability of system evolution, and pointed out the formulation of reasonable innovation income distribution scheme and effective regulation of enterprises by government departments [38]. Vaida believes that government policies and financial support are important factors affecting enterprise technological innovation [39]. Zhang constructs a tripartite evolutionary game model involving two manufacturing enterprises and the government in the monopolistic competitive market and analyzes the stability of each party's strategy selection [40].

### 2.3. Literature Gaps

Most of the above studies have examined the impact of financing and government intervention on corporate technological innovation through an empirical approach, and these studies have clarified the impact of corporate financing on corporate technological innovation and the role of government in it. However, most of these studies have focused on the impact of government intervention or a single aspect of corporate financing constraints. The interaction between government, financial institutes, and enterprises is less often discussed. There is also little literature that explores in depth the different investment options of financial institutes. This study fills this gap by analyzing the interaction mechanism between government subsidies, financial institutes' investment choices, and enterprises' R&D investment intensity from a game perspective. Both equity financing and debt financing approaches are considered.

## 3. Research Methods

### 3.1. Model Overview

Science-tech enterprises, government, and financial institutes are very important stakeholders in innovation strategies. In this study, we will use the evolutionary game to study the influence of behavior interaction between the three game agents and analyze the evolutionary stability of the system under different circumstances and the important factors affecting its evolutionary stability.

The three-party game process is shown in Figure 1.

### 3.2. Model Assumptions

  Assumption 1: suppose the three game agents of science-tech enterprises, government, and financial institutes are limited rational agents with the goal of maximizing their own interests. They will constantly adjust and improve their strategic choices according to their own benefits in the game process.
  Assumption 2: suppose the strategy of science-tech enterprises is “Innovation with High R&D Intensity” or “Innovation with Low R&D Intensity.” The government's strategy is “Subsidy” or “no Subsidy,” and the strategy of financial institutes is “Equity investment” or “Debt investment.” The R&D expense of science-tech enterprises is all funding by the external financing from financial institutes and government.
  Assumption 3: technological innovation can bring positive external economy and benefits to the government. The higher density of R & D investment in science-tech enterprises *α*, the higher economic and social externality multiplier by innovation g, so we assume *g*_*Q*_ > *g*_*L*_.
  Assumption 4: reputation multiplier by government subsidies *k*(*k* > 1) enhance the output of enterprise innovation investment.
  Assumption 5: government subsidies can share the risk of debt investment of financial institutes， so we assume *r*_*S*_ > *r*_*N*_.

### 3.3. Parameters' Setting

The parameters' setting and explanations in the model are shown in Table 1.

### 3.4. Model Construction

Science-tech enterprise, government, and financial institute make strategic choices based on self-willing. Assuming that the probability of science-tech enterprise choosing “innovation with high R & D intensity” strategy is *x*, the probability of choosing “innovation with low R & D intensity” strategy is 1 − *x*. The probability of the government choosing the “subsidy” strategy is *y*, and the probability of choosing the “no subsidy” strategy is 1 − *y*. If the probability of financial institutes choosing “equity investment” is *Z*, the probability of choosing “debt investment” is 1 − *z*. Based on above, the income matrix of the three parties is shown in Table 2.

## 4. Results and Discussion

### 4.1. Construct Expectation Function

#### 4.1.1. Enterprise Expectation Function

The expected return of enterprises' choosing strategy *Q* of “innovation with high R & D intensity” is *E*_*Q*_, the expected return of enterprises choosing strategy *L* of “innovation with low R & D intensity” is *E*_*L*_, and the average expected return $\bar{E_{I}}$ will be

(1) $$\begin{array}{c} E_{Q}=yz\left(F_{Q}+S_{Q}\right)\alpha_{Q}\beta_{Q}k+\left(1-y\right)zF_{Q}\alpha_{Q}\beta_{Q}+y\left(1-z\right)\left[\left(F_{Q}+S_{Q}\right)\alpha_{Q}\beta_{Q}k-F_{Q}\left(r_{S}+1\right)\right]+\left(1-y\right)\left(1-z\right)\left[F_{Q}\alpha_{Q}\beta_{Q}-F_{Q}\left(r_{N}+1\right)\right],\\ E_{L}=yz\left(F_{L}+S_{L}\right)\alpha_{L}\beta_{L}k+\left(1-y\right)zF_{L}\alpha_{L}\beta_{L}+y\left(1-z\right)\left[\left(F_{L}+S_{L}\right)\alpha_{L}\beta_{L}k-F_{L}\left(r_{S}+1\right)\right]+\left(1-y\right)\left(1-z\right)\left[F_{L}\alpha_{L}\beta_{L}-F_{L}\left(r_{N}+1\right)\right],\\ \bar{E_{I}}=xE_{Q}+\left(1-x\right)E_{L}. \end{array}$$

#### 4.1.2. Government Expectation Function

The expected return of government choosing “subsidy” is *E*_*S*_, the expected return of choosing “no subsidy” is *E*_*N*_, and the average expected return $\bar{E_{G}}$ will be

(2) $$\begin{array}{c} E_{S}=x\left[\left(F_{Q}+S_{Q}\right)\alpha_{Q}\beta_{Q}kg_{Q}-S_{Q}-C_{G}\right]+\left(1-x\right)\left[\left(F_{L}+S_{L}\right)\alpha_{L}\beta_{L}kg_{L}-S_{L}-C_{G}\right],\\ E_{N}=xF_{Q}\alpha_{Q}\beta_{Q}g_{Q}+\left(1-x\right)F_{L}\alpha_{L}\beta_{L}g_{L},\\ \bar{E_{G}}=yE_{S}+\left(1-y\right)E_{N}. \end{array}$$

#### 4.1.3. Financial Institute Expectation Function

The expected return of financial institute choosing “equity investment” is *E*_*E*_, the expected return of choosing “debt investment” is *E*_*D*_, and the average expected return $\bar{E_{F}}$ will be

(3) $$\begin{array}{c} E_{E}=xy\left(F_{Q}+S_{Q}\right)\alpha_{Q}\beta_{Q}k\delta +x\left(1-y\right)F_{Q}\alpha_{Q}\beta_{Q}\delta +\left(1-x\right)y\left(F_{L}+S_{L}\right)\alpha_{L}\beta_{L}k\delta +\left(1-x\right)\left(1-y\right)F_{L}\alpha_{L}\beta_{L}\delta ,\\ E_{D}=xyF_{Q}r_{S}+x\left(1-y\right)F_{Q}r_{N}+\left(1-x\right)yF_{L}r_{S}+\left(1-x\right)\left(1-y\right)F_{L}r_{N},\\ \bar{E_{F}}=zE_{E}+\left(1-z\right)E_{D}. \end{array}$$

### 4.2. Malthusian Replicated Dynamic Differential Equation Solution

The replicated dynamic differential equation for the choice of an active strategy by science-tech enterprises, government, and financial institutes can be expressed as follows:

(1) Science-tech enterprises' replicated dynamic differential equation:
  (4) $$\begin{array}{c} F\left(x\right)=\frac{dx}{dt}\\ =x\left(E_{Q}-\bar{E_{I}}\right)\\ =x\left(1-x\right)\left(E_{Q}-E_{L}\right)\\ =x\left(1-x\right)\left[\left(1+yk-y\right)\left(\alpha_{Q}\beta_{Q}F_{Q}-\alpha_{L}\beta_{L}F_{L}\right)+yk\left(\alpha_{Q}\beta_{Q}S_{Q}-\alpha_{L}\beta_{L}S_{L}\right)-\left(1-z\right)\left(yr_{S}+r_{N}+1-yr_{N}\right)\left(F_{Q}-F_{L}\right)\right]. \end{array}$$
(2) Government's replicated dynamic differential equation:
  (5) $$\begin{array}{c} F\left(y\right)=\frac{dy}{dt}\\ =y\left(E_{S}-\bar{E_{G}}\right)\\ =y\left(1-y\right)\left(E_{S}-E_{N}\right)\\ =y\left(1-y\right)\left[x\alpha_{Q}\beta_{Q}g_{Q}\left(k-1\right)F_{Q}+x\left(\alpha_{Q}\beta_{Q}g_{Q}k-1\right)S_{Q}+\left(1-x\right)\alpha_{L}\beta_{L}g_{L}\left(k-1\right)F_{L}+\left(1-z\right)\left(\alpha_{L}\beta_{L}g_{L}k-1\right)S_{L}-C_{G}\right]. \end{array}$$
(3) Financial institutes' replicated dynamic differential equation:
  (6) $$\begin{array}{c} F\left(z\right)=\frac{dz}{dt}\\ =z\left(E_{E}-\bar{E_{F}}\right)\\ =z\left(1-z\right)\left(E_{E}-E_{D}\right)\\ =z\left(1-z\right)\left\{x\left[\left(yk+1-y\right)\alpha_{Q}\beta_{Q}\delta -yr_{S}-\left(1-y\right)r_{N}\right]F_{Q}+xyk\alpha_{Q}\beta_{Q}\delta S_{Q}+\left(1-x\right)\left[\left(yk+1-y\right)\alpha_{L}\beta_{L}\delta -yr_{S}-\left(1-y\right)r_{N}\right]F_{L}+\left(1-x\right)yk\alpha_{L}\beta_{L}\delta S_{L}\right\}. \end{array}$$

Combining three equations, we will get the replication power system of science-tech enterprise, government, and financial institutes as below:

(7) $$\begin{array}{c} \left\{\begin{array}{c} F\left(x\right)=x\left(1-x\right)\left[\left(1+yk-y\right)\left(\alpha_{Q}\beta_{Q}F_{Q}-\alpha_{L}\beta_{L}S_{L}\right)-\left(1-z\right)\left(yr_{S}+r_{N}+1-yr_{N}\right)\left(F_{Q}-F_{L}\right)\right],\\ F\left(y\right)=y\left(1-y\right)\left[x\alpha_{Q}\beta_{Q}g_{Q}\left(k-1\right)F_{Q}+x\left(\alpha_{Q}\beta_{Q}g_{Q}k-1\right)S_{Q}+\left(1-x\right)\alpha_{L}\beta_{L}g_{L}\left(k-1\right)F_{L}+\left(1-z\right)\left(\alpha_{L}\beta_{L}g_{L}k-1\right)S_{L}-C_{G}\right],\\ F\left(z\right)=z\left(1-z\right)\left\{x\left[\left(yk+1-y\right)\alpha_{Q}\beta_{Q}\delta -yr_{S}-\left(1-y\right)r_{N}\right]F_{Q}+xyk\alpha_{Q}\beta_{Q}\delta S_{Q}+\left(1-x\right)\left[\left(yk+1-y\right)\alpha_{L}\beta_{L}\delta -yr_{S}-\left(1-y\right)r_{N}\right]F_{L}+\left(1-x\right)yk\alpha_{L}\beta_{L}\delta S_{L}\right\}. \end{array}\right. \end{array}$$

### 4.3. Strategy Portfolio Stability Analysis

#### 4.3.1. Equilibrium of Dynamic System

According to Takalo and Tanayama [11]，we can judge the strategy portfolio stability by analyzing the Jacobian matrix; then, we conduct the replicated dynamic system Jacobian matrix:

(8) $$\begin{array}{c} J=\left(\begin{array}{ccc} P_{11} & P_{12} & P_{13}\\ P_{21} & P_{22} & P_{23}\\ P_{31} & P_{32} & P_{33} \end{array}\right). \end{array}$$

Among them,

(9) $$\begin{array}{c} P_{11}=\frac{\partial F\left(x\right)}{\partial x}\\ =\left(1-2x\right)\left[\left(1+yk-y\right)\left(\alpha_{Q}\beta_{Q}F_{Q}-\alpha_{L}\beta_{L}F_{L}\right)+yk\left(\alpha_{Q}\beta_{Q}S_{Q}-\alpha_{L}\beta_{L}S_{L}\right)-\left(1-z\right)\left(yr_{S}+r_{N}+1-yr_{N}\right)\left(F_{Q}-F_{L}\right)\right],\\ P_{12}=\frac{\partial F\left(x\right)}{\partial y}\\ =x\left(1-x\right)\left[\left(k-1\right)\left(\alpha_{Q}\beta_{Q}F_{Q}-\alpha_{L}\beta_{L}F_{L}\right)+k\left(\alpha_{Q}\beta_{Q}S_{Q}-\alpha_{L}\beta_{L}S_{L}\right)-\left(1-z\right)\left(r_{S}-r_{N}\right){\left(F_{Q}-F\right)}_{L}\right],\\ P_{13}=\frac{\partial F\left(x\right)}{\partial z}\\ =x\left(1-x\right)\left(yr_{S}+r_{N}+1-yr_{N}\right)\left(F_{Q}-F_{L}\right),\\ P_{21}=\frac{\partial F\left(y\right)}{\partial x}\\ =y\left(1-y\right)\left[\alpha_{Q}\beta_{Q}g_{Q}\left(k-1\right)F_{Q}+\left(\alpha_{Q}\beta_{Q}g_{Q}k-1\right)S_{Q}-\alpha_{L}\beta_{L}g_{L}\left(k-1\right)F_{L}-\left(\alpha_{L}\beta_{L}g_{L}k-1\right)S_{L}\right],\\ P_{22}=\frac{\partial F\left(y\right)}{\partial y}\\ =\left(1-2y\right)\left[x\alpha_{Q}\beta_{Q}g_{Q}\left(k-1\right)F_{Q}+x\left(\alpha_{Q}\beta_{Q}g_{Q}k-1\right)S_{Q}+\left(1-x\right)\alpha_{L}\beta_{L}g_{L}\left(k-1\right)F_{L}+\left(1-z\right)\left(\alpha_{L}\beta_{L}g_{L}k-1\right)S_{L}-C_{G}\right],\\ P_{23}=\frac{\partial F\left(y\right)}{\partial z}\\ =0,\\ P_{31}=\frac{\partial F\left(z\right)}{\partial x}\\ =z\left(1-z\right)\left\{\left[\left(yk+1-y\right)\alpha_{Q}\beta_{Q}\delta -yr_{S}-\left(1-y\right)r_{N}\right]F_{Q}+yk\alpha_{Q}\beta_{Q}\delta S_{Q}-\left[\left(yk+1-y\right)\alpha_{L}\beta_{L}\delta -yr_{S}-\left(1-y\right)r_{N}\right]F_{L}-yk\alpha_{L}\beta_{L}\delta S_{L}\right\},\\ P_{32}=\frac{\partial F\left(z\right)}{\partial y}\\ =z\left(1-z\right)\left\{xF_{Q}\left[\left(k-1\right)\alpha_{Q}\beta_{Q}\delta -r_{S}+r_{N}\right]+xk\alpha_{Q}\beta_{Q}\delta S_{Q}+\left(1-z\right)F_{L}\left[\left(k-1\right)\alpha_{L}\beta_{L}\delta -r_{S}+r_{N}\right]+\left(1-z\right)k\alpha_{L}\beta_{L}\delta S_{L}\right\},\\ P_{33}=\frac{\partial F\left(z\right)}{\partial z}\\ =\left(1-2z\right)\left\{x\left[\left(yk+1-y\right)\alpha_{Q}\beta_{Q}\delta -yr_{S}-\left(1-y\right)r_{N}\right]F_{Q}+xyk\alpha_{{}_{Q}}\beta_{Q}\delta S_{Q}+\left(1-x\right)\left[\left(yk+1-y\right)\alpha_{L}\beta_{L}\delta -yr_{S}-\left(1-y\right)r_{N}\right]F_{L}+\left(1-x\right)yk\alpha_{L}\beta_{L}\delta S_{L}\right\}. \end{array}$$

In the dynamic system composed of three game agents, assuming F(*x*) = 0, F (*y*) = 0, and F (*z*) = 0, we obtain eight Nash equilibrium points of the system: O(0, 0, 0), A(0, 0, 1), B(0, 1, 0), C(0, 1, 1), D(1, 0, 0), E(1, 0, 1),F (1, 1, 0), and G(1, 1, 1).

According to Lyapunov's first law, if the eigenvalues of the corresponding matrix are all negative, the equilibrium point is the system's ESS. The stability of each point is shown in Table 3.

#### 4.3.2. Equilibrium Stability Analysis

The calculations reveal that this study should analyze the game's stabilization strategy in 8 scenarios.

Scenario 1: if the following conditions are satisfied, the equilibrium is *G* (1, 1, 1):
  (10) $$\begin{array}{c} \left\{\begin{array}{c} \alpha_{L}\beta_{L}\left(F_{L}+S_{L}\right)<\alpha_{Q}\beta_{Q}\left(F_{Q}+S_{Q}\right),\\ C_{G}<\alpha_{Q}\beta_{Q}g_{Q}\left(k-1\right)F_{Q}+\left(\alpha_{Q}\beta_{Q}g_{Q}k-1\right)S_{Q},\\ r_{S}F_{Q}<k\alpha_{Q}\beta_{Q}\delta \left(S_{Q}+F_{Q}\right). \end{array}\right. \end{array}$$
When *α*_*L*_*β*_*L*_(*F*_*L*_+*S*_*L*_) < *α*_*Q*_*β*_*Q*_(*F*_*Q*_+*S*_*Q*_), *C*_*G*_ < *α*_*Q*_*β*_*Q*_*g*_*Q*_(*k* − 1)*F*_*Q*_+(*α*_*Q*_*β*_*Q*_*g*_*Q*_*k* − 1)*S*_*Q*_, *r*_*S*_*F*_*Q*_ < *kα*_*Q*_*β*_*Q*_*δ*(*S*_*Q*_+*F*_*Q*_), the eigenvalues of the Jacobi matrix corresponding to the evolutionary stability point G(1, 1, 1) are negative, indicating that G(1, 1, 1) is ESS. This indicates that science-tech enterprises choose high R&D intensity when the benefits from innovation investment of high R&D intensity firms exceeds that of low R&D intensity firms. When the socio-economic benefits increased by government subsidies outweigh the administrative costs, the government chooses to implement subsidies for high R&D-intensive enterprises. Therefore, financial institutes choose to make equity investments when the return on equity investment in high R&D intensity enterprises that receive government subsidies is greater than the return on debt investment.
Scenario 2: if the following conditions are satisfied, the equilibrium is F (1, 1, 0):
  (11) $$\begin{array}{c} \left\{\begin{array}{c} k\alpha_{L}\beta_{L}\left(F_{L}+S_{L}\right)+\left(r_{S}+1\right)\left(F_{Q}-F_{L}\right)<k\alpha_{Q}\beta_{Q}\left(F_{Q}+S_{Q}\right),\\ C_{G}<\alpha_{Q}\beta_{Q}g_{Q}\left(k-1\right)F_{Q}+\left(\alpha_{Q}\beta_{Q}g_{Q}k-1\right)S_{Q},\\ k\alpha_{Q}\beta_{Q}\delta \left(S_{Q}+F_{Q}\right)<r_{S}F_{Q}. \end{array}\right. \end{array}$$
When *kα*_*L*_*β*_*L*_(*F*_*L*_+*S*_*L*_)+(*r*_*S*_+1)(*F*_*Q*_ − *F*_*L*_) < *kα*_*Q*_*β*_*Q*_(*F*_*Q*_+*S*_*Q*_), *C*_*G*_ < *α*_*Q*_*β*_*Q*_*g*_*Q*_(*k* − 1)*F*_*Q*_+(*α*_*Q*_*β*_*Q*_*g*_*Q*_*k* − 1)*S*_*Q*_, and *kα*_*Q*_*β*_*Q*_*δ*(*S*_*Q*_+*F*_*Q*_) < *r*_*S*_*F*_*Q*_, the eigenvalues of the Jacobi matrix corresponding to the evolutionary stability point F (1, 1, 0) are negative, indicating that F (1, 1, 0) is ESS. This indicates that enterprises choose a high R&D intensity when the total benefits termed by the high R&D intensity technology are higher than those received by the low R&D intensity firm. The total benefits include the subsidies received from the government and the resulting reputational value added (this reputational value added mainly comes in the form of obtaining lower debt financing costs). The government will choose to subsidize high R&D intensity enterprises when the socio-economic benefits of government subsidies outweigh the administrative costs. Financial institutes, on the contrary, have a greater return on debt investment than on equity investment and therefore choose debt investment.
Scenario 3: if the following conditions are satisfied, the equilibrium is E (1, 0, 1):
  (12) $$\begin{array}{c} \left\{\begin{array}{c} \alpha_{L}\beta_{L}F_{L}<\alpha_{Q}\beta_{Q}F_{Q},\\ \alpha_{Q}\beta_{Q}g_{Q}\left(k-1\right)F_{Q}+\left(\alpha_{Q}\beta_{Q}g_{Q}k-1\right)S_{Q}<C_{G},\\ r_{N}<\alpha_{Q}\beta_{Q}\delta . \end{array}\right. \end{array}$$
When *α*_*L*_*β*_*L*_*F*_*L*_ < *α*_*Q*_*β*_*Q*_*F*_*Q*_, *α*_*Q*_*β*_*Q*_*g*_*Q*_(*k* − 1)*F*_*Q*_+(*α*_*Q*_*β*_*Q*_*g*_*Q*_*k* − 1)*S*_*Q*_ < *C*_*G*_, and *r*_*N*_ < *α*_*Q*_*β*_*Q*_*δ*, the eigenvalues of the Jacobi matrix corresponding to the evolutionary stability point *E* (1, 0, 1) are negative, indicating that *E* (1, 0, 1) is ESS. This indicates that enterprises that receive equity investment from financial institutes for high R&D intensity will choose high R&D intensity when the return is greater than the return for low R&D intensity. The government will not subsidize when the economic and social benefits gained from government subsidies are not sufficient to offset the cost of administration. Financial institutes choose to make equity investments in high R&D intensity enterprises when the rate of return on equity investments in science-tech enterprises is greater than that of return on debt investments.
Scenario 4: if satisfy the following conditions, the equilibrium is D (1, 0, 0):
  (13) $$\begin{array}{c} \left\{\begin{array}{c} \alpha_{L}\beta_{L}F_{L}+\left(r_{N}+1\right)\left(F_{Q}-F_{L}\right)<\alpha_{Q}\beta_{Q}F_{Q},\\ \alpha_{Q}\beta_{Q}g_{Q}\left(k-1\right)F_{Q}+\left(\alpha_{Q}\beta_{Q}g_{Q}k-1\right)S_{Q}<C_{G},\\ \alpha_{Q}\beta_{Q}\delta <r_{N}. \end{array}\right. \end{array}$$
When *α*_*L*_*β*_*L*_*F*_*L*_+(*r*_*N*_+1)(*F*_*Q*_ − *F*_*L*_) < *α*_*Q*_*β*_*Q*_*F*_*Q*_, *α*_*Q*_*β*_*Q*_*g*_*Q*_(*k* − 1)*F*_*Q*_+(*α*_*Q*_*β*_*Q*_*g*_*Q*_*k* − 1)*S*_*Q*_ < *C*_*G*_, and *α*_*Q*_*β*_*Q*_*δ* < *r*_*N*_, the eigenvalues of the Jacobi matrix corresponding to the evolutionary stability point D (1, 0, 0) are negative, indicating that D (1, 0, 0) is ESS. This indicates that enterprises that receive loans from financial institutes will choose high R&D intensity when the return of innovation investment for high R&D intensity is greater than the return for low R&D intensity. The government subsidizes when the economic and social benefits gained from government subsidies are not sufficient to offset the cost of administration. Financial institutes choose to make debt investments in high R&D intensity enterprises when the return on equity investment in science-tech enterprises is less than the return on debt investment.
Scenario 5: if the following conditions are satisfied, the equilibrium is C (0, 1, 1):
  (14) $$\begin{array}{c} \left\{\begin{array}{c} \alpha_{Q}\beta_{Q}\left(F_{Q}+S_{Q}\right)<\alpha_{L}\beta_{L}\left(F_{L}+S_{L}\right),\\ C_{G}<\alpha_{L}\beta_{L}g_{L}\left(k-1\right)F_{L}+\left(\alpha_{L}\beta_{L}g_{L}k-1\right)S_{L},\\ r_{S}F_{L}<k\alpha_{L}\beta_{L}\delta \left(S_{L}+F_{L}\right). \end{array}\right. \end{array}$$
When *α*_*Q*_*β*_*Q*_(*F*_*Q*_+*S*_*Q*_) < *α*_*L*_*β*_*L*_(*F*_*L*_+*S*_*L*_), *C*_*G*_ < *α*_*L*_*β*_*L*_*g*_*L*_(*k* − 1)*F*_*L*_+(*α*_*L*_*β*_*L*_*g*_*L*_*k* − 1)*S*_*L*_, and *r*_*S*_*F*_*L*_ < *kα*_*L*_*β*_*L*_*δ*(*S*_*L*_+*F*_*L*_), the eigenvalues of the Jacobi matrix corresponding to the evolutionary stability point C (0, 1, 1) are negative, indicating that C (0, 1, 1) is ESS. This indicates that the enterprises choose to make low R&D intensity, when the benefits of high R&D intensity are less than the benefits of low R&D intensity. The government chooses to subsidize when the economic and social benefits gained from government subsidies outweigh the administrative costs. Financial institutes choose to make equity investments in low R&D intensity enterprises when the return on equity investment in low R&D intensity science-tech enterprises is greater than the return on debt investment. Science-tech enterprises receive government subsidies and equity financing to invest in R&D.
Scenario 6: if the following conditions are satisfied, the equilibrium is B(0, 1, 0):
  (15) $$\begin{array}{c} \left\{\begin{array}{c} k\alpha_{Q}\beta_{Q}\left(F_{Q}+S_{Q}\right)-\left(r_{S}+1\right)\left(F_{Q}-F_{L}\right)<k\alpha_{L}\beta_{L}\left(F_{L}+S_{L}\right),\\ C_{G}<\alpha_{L}\beta_{L}g_{L}\left(k-1\right)F_{L}+\left(\alpha_{L}\beta_{L}g_{L}k-1\right)S_{L},\\ k\alpha_{L}\beta_{L}\delta \left(S_{L}+F_{L}\right)<r_{S}F_{L}. \end{array}\right. \end{array}$$
When *kα*_*Q*_*β*_*Q*_(*F*_*Q*_+*S*_*Q*_) − (*r*_*S*_+1)(*F*_*Q*_ − *F*_*L*_) < *kα*_*L*_*β*_*L*_(*F*_*L*_+*S*_*L*_), *C*_*G*_ < *α*_*L*_*β*_*L*_*g*_*L*_(*k* − 1)*F*_*L*_+(*α*_*L*_*β*_*L*_*g*_*L*_*k* − 1)*S*_*L*_, and *kα*_*L*_*β*_*L*_*δ*(*S*_*L*_+*F*_*L*_) < *r*_*S*_*F*_*L*_, the eigenvalues of the Jacobi matrix corresponding to the evolutionary stability point B (0, 1, 0) are negative, indicating that B (0, 1, 0) is ESS. This indicates that the enterprises choose low R&D intensity, when the benefits of high R&D intensity are less than the benefits obtained from low R&D intensity. The government chooses to subsidize when the economic and social benefits gained from government subsidies outweigh the administrative costs. Financial institutes choose to make debt investments in low R&D intensity enterprises when the return on equity investment is less than the return on debt investment. Science-tech enterprises receive government subsidies and debt financing for R&D investment.
Scenario 7: if the following conditions are satisfied, the equilibrium is A (0, 0, 1):
  (16) $$\begin{array}{c} \left\{\begin{array}{c} \alpha_{Q}\beta_{Q}F_{Q}<\alpha_{L}\beta_{L}F_{L},\\ \alpha_{L}\beta_{L}g_{L}\left(k-1\right)F_{L}+\left(\alpha_{L}\beta_{L}g_{L}k-1\right)S_{L}<C_{G},\\ r_{N}<\alpha_{L}\beta_{L}\delta . \end{array}\right. \end{array}$$
When *α*_*Q*_*β*_*Q*_*F*_*Q*_ < *α*_*L*_*β*_*L*_*F*_*L*_, *α*_*L*_*β*_*L*_*g*_*L*_(*k* − 1)*F*_*L*_+(*α*_*L*_*β*_*L*_*g*_*L*_*k* − 1)*S*_*L*_ < *C*_*G*_, and *r*_*N*_ < *α*_*L*_*β*_*L*_*δ*, the eigenvalues of the Jacobi matrix corresponding to the evolutionary stability point A (0, 0, 1) are negative, indicating that A (0, 0, 1) is ESS. This indicates that enterprises choose low R&D intensity when the return of innovation investment is less. The government will not subsidize when the economic and social benefits gained are not sufficient to offset the cost of administration. Financial institutes choose to make equity investments in low R&D intensity enterprises when the return is greater than that on debt investment.
Scenario 8: if the following conditions are satisfied, the equilibrium is O (0, 0, 0):
  (17) $$\begin{array}{c} \left\{\begin{array}{c} \alpha_{Q}\beta_{Q}F_{Q}-\left(r_{N}+1\right)\left(F_{Q}-F_{L}\right)<\alpha_{L}\beta_{L}F_{L},\\ \alpha_{L}\beta_{L}g_{L}\left(k-1\right)F_{L}+\left(\alpha_{L}\beta_{L}g_{L}k-1\right)S_{L}<C_{G},\\ \alpha_{L}\beta_{L}\delta <r_{N}. \end{array}\right. \end{array}$$
When *α*_*Q*_*β*_*Q*_*F*_*Q*_ − (*r*_*N*_+1)(*F*_*Q*_ − *F*_*L*_) < *α*_*L*_*β*_*L*_*F*_*L*_, *α*_*L*_*β*_*L*_*g*_*L*_(*k* − 1)*F*_*L*_+(*α*_*L*_*β*_*L*_*g*_*L*_*k* − 1)*S*_*L*_ < *C*_*G*_, and *α*_*L*_*β*_*L*_*δ* < *r*_*N*_, the eigenvalues of the Jacobi matrix corresponding to the evolutionary stability point O (0, 0, 0) are negative, indicating that O (0, 0, 0) is ESS. This indicates that enterprises will choose low R&D intensity, when the profit of innovation investment is less. The government will not subsidize when the economic and social benefits gained from government subsidies are not sufficient to offset the cost of administration. Financial institutes choose debt investments in low R&D intensity enterprises when the return on equity investments is less than the return on debt investments.

Based on the above evolutionary game model, we analyze the eight scenarios of different strategy portfolios chosen by enterprises, government, and financial institutes. For the three players, one's choice is the condition which can influence other two's choices. Enterprises choose high R&D intensity instead of low R&D intensity if the output of former exceeds that of the latter. Enterprises' R&D output is closely related to the strategy choices of the government and financial institutes. The government chooses provide subsidy if its benefits exceed its costs. As the government pays attention to broad economic and social targets, the benefits include not only the R&D output itself but also economic and social externalities and the regulation effect to enterprises. The cost includes subsidies as well as administrative costs. Financial institutes make strategy choices between equity investment and debt investment based on their investment yields. The debt investment yield is different with government subsidies from that without government subsidies.

## 5. Numerical Simulation

### 5.1. The Evolutionary Trajectory of ESS

For analyzing the dynamic evolution process, the strategy evolution process of the tripartite game in different scenarios can be simulated by changing the parameter settings. In this section, different stability conditions are brought into MATLAB R2022a to simulate the evolutionary trajectory.

1. Assume *F*_*Q*_ = 100, *F*_*L*_ = 80, *α*_*Q*_ = 0.3, *α*_*L*_ = 0.2, *β*_*Q*_ = 1.5, *β*_*L*_ = 1.2, *S*_*Q*_ = 10, *S*_*L*_ = 8, *k* = 1.2, *C*_*G*_ = 1, *g*_*Q*_ = 1.2, *g*_*L*_ = 1.1, *δ* = 0.3, *r*_*S*_ = 0.05, and *r*_*N*_ = 0.08. The evolutionary trajectory of *G* (1, 1, 1) is featured in Figure 2(a). When the initial probabilities of all three parties are 0.4, the evolutionary trajectory is displayed in Figure 2(b).
2. Assume *F*_*Q*_ = 100, *F*_*L*_ = 80, *α*_*Q*_ = 0.3, *α*_*L*_ = 0.2, *β*_*Q*_ = 1.5, *β*_*L*_ = 1.2, *S*_*Q*_ = 10, *S*_*L*_ = 8, *k* = 1.2, *C*_*G*_ = 1, *g*_*Q*_ = 1.2, *g*_*L*_ = 1.1, *δ* = 0.1, *r*_*S*_ = 0.06, and *r*_*N*_ = 0.08. The evolutionary trajectory of F (1, 1, 0) is featured in Figure 3(a). When the initial probabilities of all three parties are 0.4, the evolutionary trajectory is displayed in Figure 3(b).
3. Assume *F*_*Q*_ = 100, *F*_*L*_ = 80, *α*_*Q*_ = 0.3, *α*_*L*_ = 0.2, *β*_*Q*_ = 1.5, *β*_*L*_ = 1.2, *S*_*Q*_ = 10, *S*_*L*_ = 8, *k* = 1.1, *C*_*G*_ = 1, *g*_*Q*_ = 1.1, *g*_*L*_ = 1.05, *δ* = 0.3, *r*_*S*_ = 0.06, and *r*_*N*_ = 0.08. The evolutionary trajectory of *E* (1, 0, 1) is featured in Figure 4(a). When the initial probabilities of all three parties are 0.4, the evolutionary trajectory is displayed in Figure 4(b).
4. Assume *F*_*Q*_ = 100, *F*_*L*_ = 80, *α*_*Q*_ = 0.3, *α*_*L*_ = 0.2, *β*_*Q*_ = 1.5, *β*_*L*_ = 1.2, *S*_*Q*_ = 10, *S*_*L*_ = 8, *k* = 1.1, *C*_*G*_ = 1, *g*_*Q*_ = 1.1, *g*_*L*_ = 1.05, *δ* = 0.1, *r*_*S*_ = 0.06, and *r*_*N*_ = 0.08. The evolutionary trajectory of D (1, 0, 0) is featured in Figure 5(a). When the initial probabilities of all three parties are 0.4, the evolutionary trajectory is displayed in Figure 5(b).
5. Assume *F*_*Q*_ = 100, *F*_*L*_ = 95, *α*_*Q*_ = 0.3, *α*_*L*_ = 0.2, *β*_*Q*_ = 1.05, *β*_*L*_ = 1.7, *S*_*Q*_ = 10, *S*_*L*_ = 8, *k* = 1.2, *C*_*G*_ = 1, *g*_*Q*_ = 1.2, *g*_*L*_ = 1.1, *δ* = 0.3, *r*_*S*_ = 0.05, and *r*_*N*_ = 0.08. The evolutionary trajectory of C (0, 1, 1) is featured in Figure 6(a). When the initial probabilities of all three parties are 0.4, the evolutionary trajectory is displayed in Figure 6(b).
6. Assume *F*_*Q*_ = 100, *F*_*L*_ = 95, *α*_*Q*_ = 0.3, *α*_*L*_ = 0.2, *β*_*Q*_ = 1.05, *β*_*L*_ = 1.7, *S*_*Q*_ = 10, *S*_*L*_ = 8, *k* = 1.2, *C*_*G*_ = 1, *g*_*Q*_ = 1.2, *g*_*L*_ = 1.1, *δ* = 0.1, *r*_*S*_ = 0.06, and *r*_*N*_ = 0.08. The evolutionary trajectory of B (0, 1, 0) is featured in Figure 7(a). When the initial probabilities of all three parties are 0.4, the evolutionary trajectory is displayed in Figure 7(b).
7. Assume *F*_*Q*_ = 100, *F*_*L*_ = 95, *α*_*Q*_ = 0.3, *α*_*L*_ = 0.2, *β*_*Q*_ = 1.05, *β*_*L*_ = 1.7, *S*_*Q*_ = 10, *S*_*L*_ = 8, *k* = 1.1, *C*_*G*_ = 1, *g*_*Q*_ = 1.1, *g*_*L*_ = 1.05, *δ* = 0.3, *r*_*S*_ = 0.06, and *r*_*N*_ = 0.07. The evolutionary trajectory of A (0, 0, 1) is featured in Figure 8(a). When the initial probabilities of all three parties are 0.4, the evolutionary trajectory is displayed in Figure 8(b).
8. Assume *F*_*Q*_ = 100, *F*_*L*_ = 95, *α*_*Q*_ = 0.3, *α*_*L*_ = 0.2, *β*_*Q*_ = 1.05, *β*_*L*_ = 1.7, *S*_*Q*_ = 10, *S*_*L*_ = 8, *k* = 1.1, *C*_*G*_ = 1, *g*_*Q*_ = 1.1, *g*_*L*_ = 1.05, *δ* = 0.1, *r*_*S*_ = 0.06, and *r*_*N*_ = 0.08. The evolutionary trajectory of O (0, 0, 0) is featured in Figure 9(a). When the initial probabilities of all three parties are 0.4, the evolutionary trajectory is displayed in Figure 9(b).

### 5.2. Single-Factor Sensitivity Analysis

#### 5.2.1. Impact of Reputation Multiplier by Government Subsidies

To evaluate the impact of reputation multiplier “*k*” by government subsidies on the evolutionary outcomes and trajectories of the innovation tripartite ESS, numerical simulations were conducted in this study. Set the initial parameters as follows. F (1, 1, 0): *F*_*Q*_ = 100, *F*_*L*_ = 80, *α*_*Q*_ = 0.3, *α*_*L*_ = 0.2, *β*_*Q*_ = 1.5, *β*_*L*_ = 1.2, *S*_*Q*_ = 10, *S*_*L*_ = 8, *k* = 1.2, *C*_*G*_ = 1, *g*_*Q*_ = 1.2, *g*_*L*_ = 1.1, *δ* = 0.1, *r*_*S*_ = 0.06, and *r*_*N*_ = 0.08.

Let *k*=1.6, 1.4, 1.2, 1.1, 1 and keep other parameters constant; the evolutionary outcomes and trajectories of tripartite ESS are as shown in Figures 10(a)–10(c). This indicates that the size of the reputation multiplier from government subsidies does not affect the R&D intensity of science-tech enterprises. This means that enterprises will choose to invest in high R&D regardless of whether government subsidies send a positive signal to the market. As the reputation multiplier from government financial subsidies increases for enterprises, the government is more willing to provide subsidies to enterprises. However, for financial institutes, the reputation multiplier from government subsidies affects the investment decisions of financial institutes. As the reputation multiplier decreases, financial institutes will be more inclined to invest in debt and will accelerate the rate of evolution.

#### 5.2.2. Impact of Economic and Social Externality Multiplier by Innovation

To evaluate the impact of economic and social externality multiplier “*g*_*Q*_” by innovation of enterprises with high R&D intensity on the evolutionary outcomes and trajectories of the innovation tripartite ESS, numerical simulations were conducted in this study. Set the initial parameters as follows. F (1, 1, 0): *F*_*Q*_ = 100, *F*_*L*_ = 80, *α*_*Q*_ = 0.3, *α*_*L*_ = 0.2, *β*_*Q*_ = 1.5, *β*_*L*_ = 1.2, *S*_*Q*_ = 10, *S*_*L*_ = 8, *k* = 1.2, *C*_*G*_ = 1, *g*_*Q*_ = 1.2, *g*_*L*_ = 1.1, *δ* = 0.1, *r*_*S*_ = 0.06, and *r*_*N*_ = 0.08.

Let *g*_*Q*_ = 1.4, 1.2, 1.1, 1, 0.9 and keep other parameters constant; the evolutionary outcomes and trajectories of tripartite ESS are as shown in Figures 11(a)–11(c). This indicates that, as the economic and social externalities from innovation by high R&D intensity enterprises increase, the government is more willing to subsidize enterprises, and enterprises are more willing to choose high R&D intensity. In contrast, a negative economic and social externality from a firm's innovation, i.e., a multiplier less than 1, increases the probability that the government will choose not to subsidize and that it will accelerate the rate of evolution. However, regardless of whether the socio-economic externality is positive or negative, financial institutes tend to choose debt investment to protect against risk.

#### 5.2.3. Impact of Revenue per Unit R&D Expense for Enterprises with High R&D Intensity

To evaluate the impact of revenue per unit R&D expense for enterprises with high R&D intensity “*β*_*Q*_” on the evolutionary outcomes and trajectories of the innovation tripartite ESS, numerical simulations were conducted in this study. Set the initial parameters as follows. F (1, 1, 0): *F*_*Q*_ = 100, *F*_*L*_ = 80, *α*_*Q*_ = 0.3, *α*_*L*_ = 0.2, *β*_*Q*_ = 1.5, *β*_*L*_ = 1.2, *S*_*Q*_ = 10, *S*_*L*_ = 8, *k* = 1.2, *C*_*G*_ = 1, *g*_*Q*_ = 1.2, *g*_*L*_ = 1.1, *δ* = 0.1, *r*_*S*_ = 0.06, and *r*_*N*_ = 0.08.

Let *β*_*Q*_ = 2, 1.8, 1.5, 1.1, 1 and keep other parameters constant; the evolutionary outcomes and trajectories of tripartite ESS are as shown in Figures 12(a)–12(c). This indicates that science-tech enterprises are more inclined to high R&D intensity as the revenue per unit of R&D expense for enterprises with high R&D intensity, and vice versa. The probability of government subsidies also increases with the revenue per unit of R&D expense for enterprises with high R&D intensity increases. Financial institutes increase the probability of debt investment as the revenue per unit of R&D expense for enterprises with high R&D intensity decreases.

#### 5.2.4. Impact of Equity Investment Earnings as % of Revenue

To evaluate the impact of equity investment earnings as % of revenue “*δ*” for science-tech enterprises “*δ*” on the evolutionary outcomes and trajectories of the innovation tripartite ESS, numerical simulations were conducted in this study. Set the initial parameters as follows. F (1, 1, 0): *F*_*Q*_ = 100, *F*_*L*_ = 80, *α*_*Q*_ = 0.3, *α*_*L*_ = 0.2, *β*_*Q*_ = 1.5, *β*_*L*_ = 1.2, *S*_*Q*_ = 10, *S*_*L*_ = 8, *k* = 1.2, *C*_*G*_ = 1, *g*_*Q*_ = 1.2, *g*_*L*_ = 1.1, *δ* = 0.1, *r*_*S*_ = 0.06, and *r*_*N*_ = 0.08.

Let *δ* = 0.05, 0.1, 0.2, 0.3, 0.4 and keep other parameters constant; the evolutionary outcomes and trajectories of tripartite ESS are as shown in Figures 13(a)–13(c). This indicates that the probability of choice by firms and government is not affected by equity investment earnings as % of revenue. Regardless of the return on equity investment, science-tech enterprises will tend to choose high R&D intensity, while the government will tend to choose subsidies. However, as the rate of return on equity investment increases, financial institutes will increase the probability of making equity investments in science-tech enterprises.

## 6. Conclusion

This study focuses on the tripartite decision-making mechanism between government, financial institutes, and technology companies on subsidies, investment patterns, and R&D intensity. The following conclusions are drawn from the study in this paper.

First, enterprises can attract government subsidy by boosting economic and social externalities. The higher density of R & D investment in the science-tech enterprises is, the higher positive external economy and benefits to the government is. As the government pays attention to broad economic and social targets, enterprises can choose the R&D projects with high positive economic and social externalities to provide incentive to the government to provide subsidy.

Second, government subsidy policy can influence the choices of enterprises and financial institutes. The government subsidies to enterprises with high R&D intensity will improve the innovation output by the innovation investment and reputation multiplier. So, the government can implement subsidy policy to attract enterprises to make high-intensive R&D activity and financial institutes to make equity investment. For small high-tech startups, government subsidy can improve their reputation in the market, which can help them to raise fund in the market and find good partners and increase the R&D output efficiency. It would be a better approach for the government to improve the market credible evaluation and subsidy recognition system for high-tech companies as a way to increase their reputation multiplier. In reality, government subsidies can take many forms and tax credit, for R&D expense is a popular policy.

Third, financial institutes' strategy choice is influenced by investment yield difference and can influence enterprises' R&D intensity choices. The policymakers can boost equity investment and R&D activity by developing capital market and optimizing subsidy policy. Supporting enterprises with high R&D intensity to go listing can attract financial institutes to make equity investment and enterprises to choose high R&D intensity strategy.

The above research results provide a good reference for policymakers to develop strategies for innovation. However, some limitations of this study still exist: this study only considers the effect of government subsidy behavior on the choice of investment patterns of financial institutions and the R&D intensity of firms, without further examining the effect of other incentive approaches. At the same time, research institutes (including universities and other institutes) need to be included in the analytical framework for exploration. Thus, multiparty decisions under multiple government incentive discretionary decisions will be the next step of research.

## Figures and Tables

**Figure 1:** The three-party game process.

**Figure 2:** (a) Three-dimensional situation of evolutionary trajectory of G(1, 1, 1). (b) Two-dimensional situation of evolutionary trajectory of G(1, 1, 1).

**Figure 3:** (a) Three-dimensional situation of evolutionary trajectory of F (1, 1, 0). (b) Two-dimensional situation of evolutionary trajectory of F (1, 1, 0).

**Figure 4:** (a) Three-dimensional situation of evolutionary trajectory of E (1, 0, 1). (b) Two-dimensional situation of evolutionary trajectory of E (1, 0, 1).

**Figure 5:** (a) Three-dimensional situation of evolutionary trajectory of D (1, 0, 0). (b) Two-dimensional situation of evolutionary trajectory of D (1, 0, 0).

**Figure 6:** (a) Three-dimensional situation of evolutionary trajectory of C (0, 1, 1). (b) Two-dimensional situation of evolutionary trajectory of C (0, 1, 1).

**Figure 7:** (a) Three-dimensional situation of evolutionary trajectory of B (0, 1, 0). (b) Two-dimensional situation of evolutionary trajectory of B (0, 1, 0).

**Figure 8:** (a) Three-dimensional situation of evolutionary trajectory of A (0, 0, 1). (b) Two-dimensional situation of evolutionary trajectory of A (0, 0, 1).

**Figure 9:** (a) Three-dimensional situation of evolutionary trajectory of O (0, 0, 0). (b) Two-dimensional situation of evolutionary trajectory of O (0, 0, 0).

**Figure 10:** Impact of the reputation multiplier by government subsidies “*k*” for (a)*k*science-tech enterprises; (b) for government; (c) for financial institutes.

**Figure 11:** Impact of economic and social externality multiplier by innovation of enterprises with high R&D intensity “*g*_*Q*_” (a) *g*_*Q*_for science-tech enterprises; (b) for government; (c) for financial institutes.

**Figure 12:** Impact of revenue per unit R&D expense for enterprises with high R&D intensity “*β*_*Q*_” (a)*β*_*Q*_for Science-Tech Enterprises; (b) for government; (c) for financial institutes.

**Figure 13:** Impact of equity investment earnings as % of revenue “*δ*” (a)*δ*for science-tech enterprises; (b) for government; (c) for financial institutes.

**Table 1:** Parameter setting and explanations.

Parameters	Explanations
*F*_*Q*_	Financial institutes' investments to enterprises with high R&D intensity
*F*_*L*_	Financial institutes' investments to enterprises with low R&D intensity
*α*_*Q*_	R&D expense as % of financing for enterprises with high R&D intensity
*α*_*L*_	R&D expense as % of financing for enterprises with low R&D intensity
*β*_*Q*_	Revenue per unit R&D expense for enterprises with high R&D intensity
*β*_*L*_	Revenue per unit R&D expense for enterprises with low R&D intensity
*S*_*Q*_	Government subsidies to enterprises with high R&D intensity
*S*_*L*_	Government subsidies to enterprises with low R&D intensity
*k*	Reputation multiplier by government subsidies
*C*_*G*_	Administrative costs of government subsidies
*g*_*Q*_	Economic and social externality multiplier by innovation of enterprises with high R&D intensity
*g*_*L*_	Economic and social externality multiplier by innovation of enterprises with low R&D intensity
*δ*	Equity investment earnings as % of revenue
*r*_*S*_	Debt investment yield with government subsidies
*r*_*N*_	Debt investment yield without government subsidies
*x*	Probability of enterprises adopting high R&D intensity strategy
*y*	Probability of government adopting subsidy policy
*z*	Probability of equity investment from financial institutes

**Table 2:** Revenue matrix.

Strategy selection	Science-tech enterprises	Government	Financial institute	
			Equity investment (*z*)	Debt investment (1 − *z*)
Innovation with high/low R&D intensity	*Q*: high R&D intensity (*x*)	Subsidies (*y*)	(*F*_*Q*_+*S*_*Q*_)*α*_*Q*_*β*_*Q*_*k*(*F*_*Q*_+*S*_*Q*_)*α*_*Q*_*β*_*Q*_*kg*_*Q*_ − *S*_*Q*_ − *C*_*G*_(*F*_*Q*_+*S*_*Q*_)*α*_*Q*_*β*_*Q*_*kδ*	(*F*_*Q*_+*S*_*Q*_)*α*_*Q*_*β*_*Q*_*k* − *F*_*Q*_(*r*_*S*_+1)(*F*_*Q*_+*S*_*Q*_)*α*_*Q*_*β*_*Q*_*kg*_*Q*_ − *S*_*Q*_ − *C*_*G*_*F*_*Q*_*r*_*S*_
		No subsidies (1 − *y*)	*F*_*Q*_ *α*_*Q*_ *β*_*Q*_ *F*_*Q*_ *α*_*Q*_ *β*_*Q*_ *g*_*Q*_ *F*_*Q*_ *α*_*Q*_ *β*_*Q*_ *δ*	*F*_*Q*_ *α*_*Q*_ *β*_*Q*_ − *F*_*Q*_(*r*_*N*_+1)*F*_*Q*_*α*_*Q*_*β*_*Q*_*g*_*Q*_*F*_*Q*_*r*_*N*_
	*L*: low R&D intensity (1 − *x*)	Subsidies (*y*)	(*F*_*L*_+*S*_*L*_)*α*_*L*_*β*_*L*_*k*(*F*_*L*_+*S*_*L*_)*α*_*L*_*β*_*L*_*kg*_*L*_ − *S*_*L*_ − *C*_*G*_(*F*_*L*_+*S*_*L*_)*α*_*L*_*β*_*L*_*kδ*	(*F*_*L*_+*S*_*L*_)*α*_*L*_*β*_*L*_*k* − *F*_*L*_(*r*_*S*_+1)(*F*_*L*_+*S*_*L*_)*α*_*L*_*β*_*L*_*kg*_*L*_ − *S*_*L*_ − *C*_*G*_*F*_*L*_*r*_*S*_
		No subsidies (1 − *y*)	*F*_*L*_ *α*_*L*_ *β*_*L*_ *F*_*L*_ *α*_*L*_ *β*_*L*_ *g*_*L*_ *F*_*L*_ *α*_*L*_ *β*_*L*_ *δ*	*F*_*L*_ *α*_*L*_ *β*_*L*_ − *F*_*L*_(*r*_*N*_+1)*F*_*L*_*α*_*L*_*β*_*L*_*g*_*L*_*F*_*L*_*r*_*N*_

**Table 3:** Jacobian matrix eigenvalues.

$\begin{array}{c} \text{Equalization }\\ \text{points} \end{array}$	Eigenvalues *λ*_1_	Eigenvalues *λ*_2_	Eigenvalues *λ*_3_
0(0,0,0)	*α*_*Q*_ *β*_*Q*_ *F*_*Q*_ − *α*_*L*_*β*_*L*_*F*_*L*_ − (*r*_*N*_+1)(*F*_*Q*_ − *F*_*L*_)	*α*_*L*_ *β*_*L*_ *g*_*L*_(*k* − 1)*F*_*L*_+(*α*_*L*_*β*_*L*_*g*_*L*_*k* − 1)*S*_*L*_ − *C*_*G*_	(*α*_*L*_*β*_*L*_*δ* − *r*_*N*_)*F*_*L*_
*A*(0,0,1)	*α*_*Q*_ *β*_*Q*_ *F*_*Q*_ − *α*_*L*_*β*_*L*_*F*_*L*_	*α*_*L*_ *β*_*L*_ *g*_*L*_(*k* − 1)*F*_*L*_+(*α*_*L*_*β*_*L*_*g*_*L*_*k* − 1)*S*_*L*_ − *C*_*G*_	(*r*_*N*_ − *α*_*L*_*β*_*L*_*δ*)*F*_*L*_
*B*(0,1,0)	*kα*_*Q*_ *β*_*Q*_(*F*_*Q*_+*S*_*Q*_) − *kα*_*L*_*β*_*L*_(*F*_*L*_+*S*_*L*_) − (*r*_*S*_+1)(*F*_*Q*_ − *F*_*L*_)	−*α*_*L*_*β*_*L*_*g*_*L*_(*k* − 1)*F*_*L*_ − (*α*_*L*_*β*_*L*_*g*_*L*_*k* − 1)*S*_*L*_+*C*_*G*_	*kα*_*L*_ *β*_*L*_ *δ*(*F*_*L*_+*S*_*L*_) − *r*_*S*_*F*_*L*_
*C*(0,1,1)	*kα*_*Q*_ *β*_*Q*_(*F*_*Q*_+*S*_*Q*_) − *kα*_*L*_*β*_*L*_(*F*_*L*_+*S*_*L*_)	−*α*_*L*_*β*_*L*_*g*_*L*_(*k* − 1)*F*_*L*_ − (*α*_*L*_*β*_*L*_*g*_*L*_*k* − 1)*S*_*L*_+*C*_*G*_	−*kα*_*L*_*β*_*L*_*δ*(*F*_*L*_+*S*_*L*_)+*r*_*S*_*F*_*L*_
*D*(1,0,0)	*α*_*L*_ *β*_*L*_ *F*_*L*_ − *α*_*Q*_*β*_*Q*_*F*_*Q*_+(*r*_*N*_+1)(*F*_*Q*_ − *F*_*L*_)	*α*_*Q*_ *β*_*Q*_ *g*_*Q*_(*k* − 1)*F*_*Q*_+(*α*_*Q*_*β*_*Q*_*g*_*Q*_*k* − 1)*S*_*Q*_ − *C*_*G*_	(*α*_*Q*_*β*_*Q*_*δ* − *r*_*N*_)*F*_*Q*_
*E*(1,0,1)	*α*_*L*_ *β*_*L*_ *F*_*L*_ − *α*_*Q*_*β*_*Q*_*F*_*Q*_	*α*_*Q*_ *β*_*Q*_ *g*_*Q*_(*k* − 1)*F*_*Q*_+(*α*_*Q*_*β*_*Q*_*g*_*Q*_*k* − 1)*S*_*Q*_ − *C*_*G*_	−(*α*_*Q*_*β*_*Q*_*δ* − *r*_*N*_)*F*_*Q*_
*F*(1,1,0)	*kα*_*L*_ *β*_*L*_(*F*_*L*_+*S*_*L*_)+(*r*_*S*_+1)(*F*_*Q*_ − *F*_*L*_) − *kα*_*Q*_*β*_*Q*_(*F*_*Q*_+*S*_*Q*_)	−[*α*_*Q*_*β*_*Q*_*g*_*Q*_(*k* − 1)*F*_*Q*_+(*α*_*Q*_*β*_*Q*_*g*_*Q*_*k* − 1)*S*_*Q*_ − *C*_*G*_]	*kα*_*Q*_ *β*_*Q*_ *δ*(*F*_*Q*_+*S*_*Q*_) − *r*_*S*_*F*_*Q*_
*G*(1,1,1)	*kα*_*L*_ *β*_*L*_(*F*_*L*_+*S*_*L*_) − *kα*_*Q*_*β*_*Q*_(*F*_*Q*_+*S*_*Q*_)	−[*α*_*Q*_*β*_*Q*_*g*_*Q*_(*k* − 1)*F*_*Q*_+(*α*_*Q*_*β*_*Q*_*g*_*Q*_*k* − 1)*S*_*Q*_ − *C*_*G*_]	*r*_*S*_ *F*_*Q*_ − *kα*_*Q*_*β*_*Q*_*δ*(*F*_*Q*_+*S*_*Q*_)

## Data Availability

All the data used to support the findings of this study are available from the corresponding author upon request.
